# Preputial skin free graft as dorsal onlay urethroplasty: Our experience of 73 patients

**DOI:** 10.4103/0970-1591.36706

**Published:** 2007

**Authors:** Shivadeo S. Bapat, Abhijit S. Padhye, Pushkaraj B. Yadav, Ashish A. Bhave

**Affiliations:** Dr. YG Bodhe Dept of Urology, Maharashtra Medical Foundation's Ratna Memorial Hospital, 986 Senapati Bapat Road, Pune - 411 004, India

**Keywords:** Dorsal onlay urethroplasty

## Abstract

**Objective:**

To present the outcome of dorsal onlay urethroplasty in 73 patients for stricture urethra over a period of eight years.

**Materials and Methods:**

Seventy-three patients of stricture urethra have undergone dorsal onlay urethroplasty from July 1998 to February 2006. Age distribution: 14-58 years. Etiology: Trauma 20/73 (27.39%), Balanitis Xerotica Obliterans 2/73 (2.73%), Iatrogenic 26/73(35.61%), Infection 3/73 (4.10%), Idiopathic 22/73 (30.13%). Site: Penobulbar-25/73, bulbar-38/73, membranous-8/73 and long length-2/73. Suprapubic catheter was inserted preoperatively: 21/73 patients. Preputial / distal penile skin was used in all patients. Buccal mucosa was not used in any patient. Hospitalization was for four to five days. Catheter was removed after 21 days. All patients had their first endoscopic checkup after three months. Subsequently they were followed up by uroflometry. Routine imaging of urethra for follow-up was not carried out.

**Results:**

63/73 (86.30%) patients had satisfactory outcome not requiring any further treatment, 8/73 (10.95%) developed anastomotic stricture (3/8-optical internal urethrotomy, 5/8 dilatation alone). 2/73 (2.75%) developed external meatal stenosis. None had urinary fistula and required repeat urethroplasty. Follow-up ranged from three months to eight years.

**Conclusion:**

Dorsal onlay urethroplasty using preputial/distal penile skin is a satisfactory procedure. Preputial/distal penile skin is devoid of hair and fat and hence an ideal graft material. Even in circumscribed patients distal penile skin can be harvested. Long-term follow-up is required in judging results of patients with stricture urethra.

Urethral stricture is a chronic and common urological problem. The principle of stricture management is to “Dilate the stricture and keep it permanently dilated”. The first part is easy but the second part poses a big challenge to urologists. Excision of strictures and primary end-to-end anastomosis can be done only in those patients with stricture length 1.5 cm or less. Where the strictures are long and more than 1.5 cm, substitution urethroplasty becomes the treatment of choice. Since *Devine*[1] in 1963 described the use of full-thickness skin graft for urethral reconstruction, there have been other innovative materials for use for urethral substitution. Naturally, the scrotal and penile skin, being very close to the urethra, has been used for urethral reconstruction.[2,3] The drawback of scrotal skin is its potential to cause intraurethral hair growth, anastomotic stricture and diverticula formation. For patients who are not circumcised prepucial skin can be utilized. Bladder epithelium harvested via a suprapubic cystostomy (SPC) has been utilized for urethral reconstruction, however, the process of harvesting the epithelia is cumbersome.[4] *Humby*[5] was the first person to describe buccal mucosa grafting in 1941 but the procedure became widely used in the 1990s and onwards.[6] Of late there have been reports that are actually advocating buccal mucosa to be the standard treatment for substitution urethroplasty[7] with success rates from 85-90%. We have been performing dorsal onlay urethroplasty using prepucial/ penile skin for the past eight years and would like to present our data.

## MATERIALS AND METHODS

A retrospective study was conducted at our institute of 73 stricture urethra patients undergoing dorsal onlay urethroplasties from July 1998 to February 2006. All urethroplasties were carried out by the author. Preoperative evaluation included history taking and physical examination. The possible etiology of the stricture was identified. After routine investigations, urine routine, culture and renal function test, the patients underwent urethrogram. Both ante-grade and retrograde urethrogram studies were performed to show the whole length of urethra. A total of 73 men underwent dorsal onlay urethroplasty from July 1998 to February 2006. Their mean age was 39.6 years (14-58 years). All patients underwent Barbagli's dorsal onlay urethroplasty using prepucial/penile skin graft.[8] Mean duration of symptoms was 16 months (five months to four years). Fifty-two patients presented with poor urinary stream while 21/73 patients had retention of urine with suprapubic cystostomy. Preoperative flow rate (Q max) in patients not on SPC was 7.2 ml/sec (5.5-10 ml/sec). Average length of the stricture was 3 cm (1.5-4 cm).

Procedure: Patient in lithotomy position following spinal anesthesia. Methylene blue was injected in the urethra to identify the urethral mucosa before starting the procedure. Urethra was mobilized from the penoscrotal junction to the bulbomembranous junction through a midline perineal incision. The urethra was opened dorsally at the stricture site. Incision was extended on the normal urethra for 1cm both proximal and distal to the stricture. Prepucial skin graft was then harvested. Subcoronal distal penile skin graft was used in those patients who were circumcised. A preputial/subcoronal skin incision was taken. Graft was dissected free from underlying connective tissue (length- 3-4 cm, width-2-2.5 cm). Graft was devoid of fat / hair follicle. The raw area of the graft was fixed and quilted on the cavernosal bed with the skin epithelium facing the urethra. Urethral mucosal edges were sutured to graft using 4 0 Vicryl sutures on cutting needle over a 16 no silicone catheter. Wound was closed in layers with a corrugated drain. Preputial/penile defect was sutured with 4 0 catgut. Postoperative wound evaluation and drain removal was carried out on the second postoperative day. Patients were sent home with the catheter on the fourth postoperative day. Catheter was removed after 21 days. Patients underwent uroflowmetry and check cystoscopy at three months. Subsequently they were followed by uroflometry. Imaging of the urethra was not carried out as a routine.

## RESULTS

A total of 73 men [Tables 1 and 2] aged between 14-58 years underwent dorsal onlay urethroplasty with penile/preputial skin graft from July 1998 to February 2006. All procedures were uneventful. Follow-up ranged from three months to eight years (mean 14 months). Successful outcome was seen in 63/73 (86.3%). Successful outcome of the procedure was confirmed when they satisfied the following criteria:

**Table 1:** Site

	(n=73)
Penobulbar	25
Bulbar	38
Bulbomembranous	8
Long length (6 cm)	2

**Table 2:** Etiology

	(n=73)
Trauma	20
Idiopathic	22
Iatrogenic	26
BXO	2
Infection	3

1. Check cystoscopy at three months after catheter removal confirming 100% take of the graft and patent urethral lumen
2. Good flow as narrated by patient
3. Documentation of the same by uroflowmetry
4. No recurrence of symptoms (poor flow, infection and dysuria)
5. No need for any further instrumentation

Postoperative uroflowetry (at three months) showed a Q max of 18 ml/sec(13.2- 25 ml/sec). Check cystoscopy done at three months after catheter removal showed good take of graft, no evidence of intraurethral hair growth or diverticula formation and near normal proximal urethra and bladder. Eight out of 73 (10.9%) developed poor urinary stream and were confirmed to have anastomotic strictures at cystoscopy. All recurrent strictures were detected at the distal end of the anastomotic site. Length was <5 mm. Three out of eight underwent optical internal urethrotomy. Subsequently these patients were put on self-dilatation. The remaining five out of eight required only filiform dilatation. Two of 73 (2.7%) patients developed external meatal stenosis. None of the patients had urinary fistula and required repeat urethroplasty.

## DISCUSSION

Surgical repair of bulbar urethral strictures is based on anastomotic repair of short lesions, while free grafts (penile or buccal) or pedicled flaps are suggested for longer or complex strictures. *Barbagli et al*.[8] showed dorsal placement of free skin / buccal mucosal graft on the corporal bodies and reported the advantages of better mechanical support, vascular supply and decreased incidence of urethrocele formation. Also there is less chance of fistula formation. Currently, dorsal onlay has definite advantages over ventral onlay –(1) graft fixity to cavernosal bed leading to better neovascularisation and maintenance of caliber of reconstructed urethra. Hence less chances of graft necrosis and failure.[9,10] (2) Good mechanical support of graft to corporal bodies reduces incidence of saccule formation which caused post voiding dribbling and ejaculatory failure.[6,7]

Earlier scrotal skin was used as pedicle flap but it lost favor due to problem of anastomotic stricture, diverticulum formation and delayed intraurethral hairball and stone formation.[3] Similarly, bladder mucosa harvesting is tedious and has lost favor.[4] The present choice for free graft is between preputial / penile skin and buccal mucosa. *Alsikafi et al*.[11] compared outcomes of buccal urethroplasty and penile skin graft urethroplasty and found that the overall success of penile skin graft urethoplasty was 84% with follow-up of 201 months and that of buccal mucosal urethroplasty was 87% with a follow-up period of 48 months. *Barbagli et al*. showed comparable results in single-stage hypospadias repair. Our results using penile/prepucial graft are comparable. Similarly, *Wessels* and *MC Aninch*[12] in their study reported comparable results of success after buccal mucosa and penile skin grafts (85%). The prepucial skin is devoid of hair and fat. Hence incidence of hair growth at anastomotic site was not seen. Another disastrous complication is graft necrosis either due to infection or failure of neovascularisation.[8,13] This is commonly seen with ventral onlay grafts and presents as urethro perineal fistula. Dorsal onlay grafts rarely have graft necrosis due to good secure fixity to the cavernosal bed.[5,11] This was confirmed in all 73 cases during our first follow-up endoscopy where all the grafts were seen well taken without any necrosis. Recurrences of obstructive urinary symptoms were seen in eight patients, of which three had tight anastomotic strictures and required OIU and subsequent self-dilatation. The remaining five had soft strictures and were treated with filiform dilatation and subsequent follow-up by uroflometry. *Barbagli et al*.[13,14] have demonstrated that penile skin grafts used as dorsal onlay had a tendency to deteriorate with time. In our study the average follow-up was for 14 months (three months- eight years) and we did not have any incidence of late failure or recurrence of obstructive symptoms.

## CONCLUSION

Dorsal onlay urethroplasty using preputial skin graft is easy, safe and gives success rates of 86.3% at mean follow-up of 14 months. These are comparable with the results given by buccal mucosal graft urethroplasty.[10,11,14]
